The article "Venous Thromboembolism Prevention in General Surgery: A Closed Loop Clinical Audit of Risk Assessment and Prophylaxis Adherence" was published in 2025. Journal: Cureus.

# Venous Thromboembolism Prevention in General Surgery: A Closed Loop Clinical Audit of Risk Assessment and Prophylaxis Adherence

**DOI:** 10.7759/cureus.93009

**Published:** 2025-09-23

**Authors:** Yusuf Yusuf, Ebrahim Matar, Noor Alfardan, Farah Naser

**Affiliations:** 1 Surgery, Harrogate District Hospital, Harrogate, GBR; 2 Surgery, Antrim Area Hospital, Antrim, GBR; 3 General Medicine, Ministry of Health Holdings, Manama, BHR; 4 General Practice, Northern Ireland Medical and Dental Training Agency (NIMDTA), Belfast, GBR

**Keywords:** acute pulmonary embolism, blood clots, general surgery, venous thromboembolsim, vte prophylaxis

## Abstract

Background: Venous thromboembolism (VTE) is a major preventable cause of morbidity and mortality in hospitalized patients. Despite established guidelines for risk assessment and prophylaxis, adherence can vary.

Methods: A two-cycle clinical audit was conducted on general surgery admissions at a district general hospital to assess adherence to National Institute for Health and Care Excellence (NICE) and local guidelines for VTE risk assessment, timely completion, and prescription of pharmacological and mechanical prophylaxis. Cycle 1 audited patients between February 7, 2023 and February 18, 2023 (n=54) and Cycle 2 audited patients between July 10, 2023 and July 17, 2023 (n=57). Interventions included education and feedback after the first cycle.

Results: In Cycle 1, 75.9% had a risk assessment completed at any time, and 53.7% within 24 hours. Pharmacological VTE prophylaxis was prescribed in 81.5%, and 29.6% received mechanical prophylaxis. In Cycle 2, completion improved to 93%, with 59.6% completed within 24 hours. Pharmacological prophylaxis was prescribed appropriately in 100%, but only 25% received mechanical prophylaxis.

Conclusions: The audit demonstrated significant improvement in pharmacological VTE prophylaxis prescription and risk assessment completion following targeted interventions, but mechanical prophylaxis adherence decreased slightly and remains an area for improvement. Regular audits and sustained education are essential to maintain and enhance compliance.

## Introduction

Venous thromboembolism (VTE), which includes deep vein thrombosis (DVT) and pulmonary embolism (PE), is a major but preventable cause of morbidity and mortality in hospitalized patients. In 2005, the House of Commons Health Committee estimated that VTE contributes to more than 25,000 deaths each year in the United Kingdom (UK) [1]. The financial impact of managing VTE, incorporating both direct and indirect costs, has been valued at approximately £640 million annually [2]. Hospital-acquired VTE refers to events occurring during admission or within 90 days of discharge and represents 50-60% of all cases [3].

The National Institute for Health and Care Excellence (NICE) provides guidance on VTE prevention, recommending prophylaxis for surgical patients at increased risk. This includes starting mechanical methods on admission and combining them with pharmacological measures when the risk of thrombosis outweighs bleeding concerns. Preventive strategies have proven effective in lowering the incidence of DVT and include mechanical methods (e.g., anti-embolism stockings, intermittent pneumatic compression devices) and pharmacological agents such as heparin and other anticoagulants [3]. To promote adherence, the National Health Service (NHS) mandated quarterly reporting of VTE risk assessments beginning in June 2010 [4].

The MEDENOX study demonstrated that factors such as acute infection, age over 75 years, cancer, and previous history of VTE substantially increase risk [5]. Despite clear national guidance, compliance remains variable [5,6]. A large intensive care unit (ICU) registry study involving 1.46 million patients reported that omission of prophylaxis within the first 24 hours (where no contraindication existed) was linked with a 35% increase in the odds of in-hospital mortality, highlighting the preventable harm associated with delays or omissions [7].

Ensuring timely and accurate VTE risk assessment and prescribing appropriate prophylaxis remain key elements of improving patient safety [8].

This audit reviews adherence to VTE risk assessment and prophylaxis protocols in general surgery patients over two audit cycles, with the aim of identifying deficiencies and evaluating the impact of educational interventions.

## Materials and methods

This audit was carried out in two cycles at Darlington Memorial Hospital in the North East of England, United Kingdom, and included both elective and emergency general surgery admissions. The objective was to assess adherence to the National Institute for Health and Care Excellence (NICE) and local trust guidelines on VTE assessment and prophylaxis.

Patients aged 18 years or older were eligible for inclusion, while those under 18 were excluded from the study. Individuals receiving therapeutic anticoagulation were included in the dataset; however, they were excluded from the statistical analysis when evaluating the appropriateness of pharmacological prophylaxis prescriptions. The first cycle included admissions between February 7, 2023 and February 18, 2023, and the second cycle included admissions between July 10, 2023 and July 17, 2023.

Data collected for each admission included whether a VTE risk assessment form had been completed, the timing of completion (within six hours and within 24 hours of admission), whether prophylaxis was prescribed when indicated, and whether the correct form of prophylaxis (mechanical or pharmacological) was provided in line with guidelines. Timing of completion was determined directly from the hospital’s electronic record timestamps, and prescription details were obtained from the electronic prescribing system. Data collection was performed retrospectively by the audit team using a standardized data collection form.

Following the first cycle, targeted interventions were implemented. These included structured education sessions and presentations delivered at departmental meetings attended by approximately 20-30 staff members, including consultants, registrars, junior doctors, nurses, and allied health professionals. Sessions were delivered online as part of routine audit meetings and lasted around 15-20 minutes. Content focused on the importance of timely VTE risk assessment, accurate documentation, and correct prescribing of prophylaxis according to national and local standards. Case examples from Cycle 1 were used to illustrate common errors and omissions, and team-specific feedback was provided to encourage reflection and highlight areas for improvement.

All data were analyzed descriptively, with categorical variables expressed as proportions. Comparisons between Cycle 1 and Cycle 2 were made using the Chi-square test. A p-value <0.05 was considered statistically significant.

## Results

A total of 111 patients were included across both cycles, with 54 in Cycle 1 and 57 in Cycle 2. Overall adherence to VTE prevention measures improved between the two audit periods. Risk assessment completion at any point during admission increased significantly from 75.9% (41/54) in Cycle 1 to 93% (53/57) in Cycle 2 (p = 0.026, chi-square) (Table 1). This result was statistically significant with a p-value of 0.026 (<0.05).

**Table 1:** Comparison of Audit Outcomes in VTE Risk Assessment and Pharmacological and Mechanical Prophylaxis Between Cycles VTE: Venous thromboembolism

Outcome	Cycle 1 (n=54)	Cycle 2 (n=57)	p-value (Chi-square)
Risk assessment completed at any time	41/54 (75.9%)	53/57 (93%)	0.026
Risk assessment completed within 24 hours	29/54 (53.7%)	34/57 (59.6%)	0.66
Pharmacological prophylaxis prescribed	44/54 (81.5%)	50/50 (100%)	0.004
Correct pharmacological dose given	41/44 (94.5%)	48/50 (96%)	0.883
Mechanical prophylaxis post-operation	16/54 (29.6%)	14/57 (25%)	0.699

Risk assessments completed within 24 hours of admission increased modestly from 53.7% (29/54) to 59.6% (34/57), though this change was not statistically significant (p = 0.660, chi-square).

Pharmacological prophylaxis prescription demonstrated significant improvement, rising from 81.5% (44/54) in Cycle 1 to 100% (50/50 eligible patients) in Cycle 2 (p = 0.004, chi-square). The improvement was statistically significant, with p < 0.05. It is to be noted that seven patients in Cycle 2 were deemed ineligible for pharmacological prophylaxis due to therapeutic anti-coagulation and were excluded from this analysis.

The proportion of patients prescribed the correct pharmacological dose also improved slightly, from 94.5% (41/44) to 0.96% (48/50), but this was not statistically significant (p = 0.883, chi-square).

In contrast, the use of mechanical prophylaxis following surgery remained low. Post-operative provision declined slightly from 29.6% (16/54) in Cycle 1 to 25% (14/57) in Cycle 2, with no statistically significant difference (p = 0.699, chi-square).

Among the patients in Cycle 1, 19 underwent emergency surgery, nine had elective surgery, and 26 were managed conservatively. In Cycle 2, 19 patients underwent emergency operations, six had elective surgery, and 32 were managed conservatively.

Errors in Cycle 1 included three patients prescribed incorrect pharmacological doses (due to factors such as weight or renal impairment) and 10 patients who required prophylaxis but did not receive it. In Cycle 2, all eligible patients received pharmacological prophylaxis, but compliance with mechanical prophylaxis continued to be suboptimal. 

## Discussion

This audit highlights ongoing challenges and modest improvements in VTE risk assessment and prophylaxis. Implementation of NICE and local guidelines provided a structured framework for prevention.

Following educational sessions and audit feedback, both risk assessment completion and pharmacological prophylaxis prescription showed significant improvement in Cycle 2. This aligns with findings from studies showing that structured improvement methods can effectively enhance prophylaxis adherence [9].

Pharmacological compliance reached 100% among eligible patients in Cycle 2, a notable and statistically significant increase from 81.5% in Cycle 1, indicating improved prescriber engagement. While the chosen references do not specifically examine weight- or renal-based dosing, they do support that educational interventions substantially improve correct pharmacological practice [10,11].

Mechanical prophylaxis usage, however, remained low at 25% in Cycle 2, with performance worsening despite the educational intervention. Literature highlights suboptimal compliance with mechanical methods, often due to a lack of clear protocols or oversight [12]. However, additional factors may also explain the poor uptake in this audit. Mechanical prophylaxis is largely a nursing-driven process, meaning adherence may depend more on ward routines and staffing than on prescriber education. Equipment availability and timely replacement may also have influenced practice, while patient compliance is another challenge, as devices are frequently uncomfortable and removed prematurely. These system-level and patient-related barriers likely limited the impact of the intervention, indicating that education alone is insufficient. Bozzato et al. [13] similarly reported that nearly 50% of patients eligible for prophylaxis fail to receive it even when guidelines recommend it, underscoring a persistent compliance gap. In a general internal medicine cohort, 20% of hospitalized patients received inappropriate VTE prophylaxis, with improper dosing, including delays or wrong dose, linked to higher rates of both thrombotic (6.5% vs 1.7%) and major bleeding events (19.6% vs 4.5%) compared to appropriately treated patients [14]. This reinforces the importance of appropriate and timely prescription and delivery of VTE prophylaxis.

Risk assessment within 24 hours modestly increased from 53.7% to 59.6%. Prompt assessment is associated with better prophylaxis rates, as supported by early intervention studies, though most research focuses on broad implementation rather than strictly 24-hour timing [15].

Our audit is limited by its single-center design, modest sample size, and reliance on documentation rather than the actual incidence of VTE. The sustainability of positive changes is uncertain, and our references highlight that without ongoing audit and system integration, improvements may regress [16,17]. The short duration of each audit cycle may not be representative of long-term practice and is susceptible to temporal biases.

Future quality improvement should incorporate automated prompts in electronic medical records; studies show that clinical decision support tools and CPOE alerts significantly increase prophylaxis compliance [9,16]. Embedding VTE prevention into electronic workflows is likely the most effective path to sustainable improvement.

## Conclusions

This audit demonstrates significant improvements in pharmacological VTE prophylaxis and risk assessment completion following targeted education and feedback. Mechanical prophylaxis usage remains suboptimal and should be addressed as a future priority. Sustained improvements will require ongoing audits, staff training, and system-level support to achieve consistent, guideline-compliant VTE prevention in surgical patients.
